# Clairvoyant: AdaBoost with Cost-Enabled Cost-Sensitive Classifier for Customer Churn Prediction

**DOI:** 10.1155/2022/9028580

**Published:** 2022-01-22

**Authors:** Hiren Kumar Thakkar, Ankit Desai, Subrata Ghosh, Priyanka Singh, Gajendra Sharma

**Affiliations:** ^1^Department of Computer Engineering, Marwadi University, 360003 Rajkot, Gujarat, India; ^2^Ahmedabad University, Ahmedabad, Gujarat, India; ^3^Ambient Scientific, Bangalore, Karnataka, India; ^4^Department of Computer Science and Engineering, School of Engineering and Sciences, SRM University, Amaravati 522240, Andhra Pradesh, India; ^5^School of Engineering, Department of Computer Science and Engineering, Kathmandu University, Dhulikhel, Kavre 45200, Nepal

## Abstract

Customer churn prediction is one of the challenging problems and paramount concerns for telecommunication industries. With the increasing number of mobile operators, users can switch from one mobile operator to another if they are unsatisfied with the service. Marketing literature states that it costs 5–10 times more to acquire a new customer than retain an existing one. Hence, effective customer churn management has become a crucial demand for mobile communication operators. Researchers have proposed several classifiers and boosting methods to control customer churn rate, including deep learning (DL) algorithms. However, conventional classification algorithms follow an error-based framework that focuses on improving the classifier's accuracy over cost sensitization. Typical classification algorithms treat misclassification errors equally, which is not applicable in practice. On the contrary, DL algorithms are computationally expensive as well as time-consuming. In this paper, a novel class-dependent cost-sensitive boosting algorithm called AdaBoostWithCost is proposed to reduce the churn cost. This study demonstrates the empirical evaluation of the proposed AdaBoostWithCost algorithm, which consistently outperforms the discrete AdaBoost algorithm concerning telecom churn prediction. The key focus of the AdaBoostWithCost classifier is to reduce false-negative error and the misclassification cost more significantly than the AdaBoost.

## 1. Introduction

In developing countries, smartphones play a significant role in human life, and the number of mobile operators is rapidly increasing in every technologically advanced country. By the end of 2019, several billion people subscribed to mobile services, accounting for nearly two-thirds of the global population [1]. These incessantly growing telecom operators are coming up with various value-added subscriptions to retain their loyal customers. Hence, customer retaining with the same service provider became questionable. In this fierce competitive nature of the wireless telecommunication industry, customers have unlimited freedom to migrate from one service provider to another. This phenomenon is known as churn. A few reasons for churn are dissatisfaction in services such as unattractive recharge plans, frequent call drops, insufficient bandwidth, frequent customer care calls, unreachable networks, and slow Internet speed. In general, several techniques are used to address the customer churn prediction such as statistical learning [2], machine learning [3], evolutionary optimization technique [4], and deep learning [5]. Boosting is an ensemble technique that attempts to create a robust classifier from several weak classifiers. AdaBoost (adaptive boosting) is the first successful algorithm developed for binary classification to improve accuracy. It has now become a somewhat feasible method for different kinds of boosting in machine learning paradigms. However, AdaBoost is inherently a cost-insensitive boosting algorithm; therefore, it has limited applications where costs need to be treated differently for different misclassification errors. This study is interested in attempting to mitigate the limitation.

In many real-world applications like anomaly detection scenarios such as bank loan defaulter, telecom churn prediction, fraudulent transactions in banks, domain feature retrieval [6], and rare diseases identification, the problem of cost-sensitive classification is predominant. The critical reasons for rising telecom churning are telecommunications' technological development, liberalization, and aggressive competition. In a highly competitive market, mobile operators mainly rely on incessant profits from existing loyal customers. In practice, the cost of acquiring a new customer is five to ten times higher than the cost of retaining an existing customer [7]. Increased churn rate is considered the plague in revenue generation because losing a royal customer client indicates losing revenue. Therefore, the leitmotiv of marketing strategy is now royal customer retention for the telecom industry. In many real-world applications, classification with imbalanced datasets encounters the misclassification costs of rare or minority classes which are usually more expensive than those of the majority classes, especially in telecom churn, medical diagnosis, and prognosis [8]. For effective customer churn management, it is essential to build an accurate churn prediction model.

Recently, cost-sensitive learning [9–14] has gained considerable interest. With the rapid use of ensemble classifiers to improve accuracy, this paper proposes a design of a misclassification cost-sensitive boosting algorithm as an extension of favourably voted boosting method AdaBoost. The clairvoyant study empirically evaluates the AdaBoostWithCost cost-sensitive boosting method to predict customer churn rate with higher accuracy than the fundamental AdaBoost classifier. In general, boosting is an ensemble technique that attempts to create a robust classifier from several weak classifiers. AdaBoost (adaptive boosting) is the first successful boosting algorithm developed for binary classification using this concept to achieve more accuracy. It has now become somewhat of a go-to method for different kinds of boosting in machine learning paradigms. However, AdaBoost fundamentally is not a cost-insensitive boosting algorithm; therefore, it has inherent limitations for applications where costs need to be treated differently for different misclassification errors. It is interested in attempting to mitigate this limitation. Most classification algorithms treat all kinds of misclassification errors, which may not be accurate in all applications in reality. In telecom churn rate prediction, the customer who will churn if mispredicted by the model has a severe impact on revenue perspective. Therefore, model accuracy may not be the correct measure index for real-world cost-sensitive applications. However, instead of optimizing the accuracy, the classification algorithm should then minimize the total misclassification cost. Therefore, the paper's key focus is on empirical evaluations and the proposed AdaBoostWithCost algorithm's theoretical issues to reduce the cumulative misclassification cost considerably better than the AdaBoost.

### 1.1. Cost-Sensitive Learning

Cost-sensitive learning is a type of learning that considers the misclassification costs [15]. The primary objective of this type of learning is to minimize the cumulative misclassification cost. The key difference between cost-sensitive learning and cost-insensitive learning is that cost-sensitive learning treats different misclassification errors differently. The cost of labelling a positive example as negative can be different from labelling a negative example as positive. Cost-insensitive learning does not consider misclassification costs. When researchers first confronted the variable cost issue, they entertained the cost-sensitive adjustments in binary classification settings [16]. Cost-sensitive learning is a distinct subfield of machine learning that takes the costs of prediction errors into account while training a machine learning model. One extra input, namely, the cost matrix, is supplied in the model-building phase of the classification process used to construct cost-sensitive models. When the cost matrix is used in association with boosting, it is said to be cost-sensitive boosting.

#### 1.1.1. The Problem of Class Imbalance

Today classification algorithms assume a proportionate distribution of examples in each class label, which is not always valid in practice. The data are said to suffer from a class imbalance problem when the class distributions are highly imbalanced. These datasets have a skewed class distribution, and they are also known as imbalanced classification problems. In this context, many classification learning algorithms have low predictive accuracy for the infrequent class [17]. In addition to assuming that the class distribution is balanced, most classifiers also assume that the costs of all types of misclassification error are equal. This assumption is not always valid in many real-world applications. In this situation, the predictive model developed using conventional machine learning algorithms could be biased and inaccurate. Researchers have put serious thought and significant attention to minimizing the misclassification cost instead of minimizing the errors. Therefore, in recent years, cost-sensitive learning has been a common approach to solving this class imbalance problem.

#### 1.1.2. Issue of Cost Sensitivity

Over the past few years, it has been observed that most of the classification algorithms assume the costs of all types of misclassification errors generated by a model as equal [36], which is often not the case for imbalanced classification problems. In class imbalance problems, the wrong prediction of a positive or minority class case is worse than incorrectly classifying an example from the negative or majority class. In recent years, cost-sensitive learning has drawn significant interest because of the increasing number of applications that involve costs such as customer churn prediction [18], fraud detection, and bank loan defaulter.

In Section 2, the problem of mobile operators along with the boosting algorithm AdaBoost is discussed. In Section 1.1, cost-sensitive learning is discussed along with problems and issues. The discussion is carried out on various classification algorithms and various popular cost-sensitive boosting algorithms in Section 2. Then, in Section 3, AdaBoostWithCost is proposed with a detailed algorithm, equations, and explanation. An empirical evaluation is performed in Section 4 by taking a dataset to investigate the algorithm on the synthesized data, and the result is generated. An evaluation of the AdaBoostWithCost algorithm and empirical results and visualizations are presented in Section 5.

## 2. Related Works

In recent years, there have been countless applications of machine learning [19] and reinforcement learning [20] in the diversified areas such as healthcare predictions [21], cloud resource management [22], and mobile robot navigation [23]. Moreover, a significant surge is also observed in cyber frauds, as well as the corresponding model to counter them, such as credit card fraud detection, telecom churn prediction [2–5], and detecting rare medical diseases. In the models mentioned above, classifiers are trained to handle most costly errors compared to others. Many ensemble-based classifications have been proposed to introduce the misclassification cost in cost-sensitive classifiers. In literature, various algorithms have been proposed over the past decades for cost-sensitive classification. Various authors have modified decision trees in different ways that consider different class-dependent costs. In [24], the cost-sensitive boosting framework has been proposed by the authors expected to optimize the loss function by applying cost-sensitive decision rules optimally. An adaptive cost bagging method was proposed in [25]. In the doctoral dissertation [21], a cost-sensitive tree stacking has been proposed where different decision trees are learned in this proposed method and then finally merged in such a way so that the cost function is minimized. In [26], a survey of cost-sensitive learning applications with base classifier as decision trees is demonstrated. The survey contains several types of cost-sensitive ensembles methods. The outline of the literature survey is described in Section 2.1.

### 2.1. Comparison and Discussion

This paper surveys various cost-sensitive boosting classifiers mentioned below. There are various popular cost-sensitive boosting algorithms [27] such as Boosting [28], Uboost, Cost-Uboost [29], AdaCost [30], and CostBoost [31] in addition to recently emerged algorithms such as CSE_1_, CSE_2_, CSE_3_, CSE_4_, and CSE_5_ [32]. It is to note that CSE stands for Cost-Sensitive Extension. All specified ten algorithms are compared and summarized in Table 1. Boosting is extended by the CostBoost algorithm. The Cost-Uboost classifier modified the Uboost. The discrete AdaBoost extended to CSE_1_, CSE_2_, and CSE_3_. In contrast, CSE_4_ and CSE_5_ are extensions of AdaCost. The goal of all these stipulated algorithms is to modify the weight in different ways in each iteration. As regards AdaCost [17] (AdaBoost with Cost-Sensitive Adaptation), Freund and Schapire's AdaBoost is the first attempt towards the study of the cost-sensitive boosting algorithm. AdaCost is a misclassification cost-sensitive boosting classifier, a variant of AdaBoost. AdaCost applies misclassifications cost in each round of boosting to update the training distribution. The central idea of AdaCost is to incorporate the cost and produce more advanced classifiers which can reduce the misclassification cost better than AdaBoost. CostBoost [31] is the extension of Boosting [28]. The modified version of Uboost is Cost-Uboost [29]. CSE_1_, CSE_2_, and CSE_3_ are extensions of discrete AdaBoost. On the contrary, CSE_4_ and CSE_5_ are extensions of AdaCost. All of these update the weight in algorithmic step. The following are the weight update equations for the cost-sensitive boosting classifiers [33].

Weight update equation for discrete AdaBoost is as follows:

(1) $$\begin{array}{c} Wt_{\left(j+1\right)}\left(m\right)=Wt_{j}\left(m\right)\exp\left(-\gamma \;H_{j}\left(x_{m}\right)\beta_{j}\right). \end{array}$$

Weight update equation for CSE_1_ is as follows:

(2) $$\begin{array}{c} Wt_{\left(j+1\right)}\left(m\right)=C_{\delta }Wt_{j}\left(m\right). \end{array}$$

Weight update equation for CSE_2_ is as follows:

(3) $$\begin{array}{c} Wt_{\left(j+1\right)}\left(m\right)=C_{\delta }Wt_{j}\left(m\right)\exp\left(-\gamma \;H_{j}\left(x_{m}\right)\right). \end{array}$$

Weight update equation for CSE_3_ is as follows:

(4) $$\begin{array}{c} Wt_{\left(j+1\right)}\left(m\right)=C_{\delta }Wt_{j}\left(m\right)\exp\left(-\gamma \;H_{j}\left(x_{m}\right)\beta_{j}\right). \end{array}$$

In AdaBoost, there is no misclassification cost included in the reweighting step. However, the misclassification cost is incorporated in the weight update equation of some cost-sensitive classifiers such as AdaCost, CSE_4_, and CSE_5_. The symbols defined in the weight update equations (1)–(3) and (4) are specified as follows. *C*_*δ*_ = cost of classification and *β*_*j*_=(1/2)ln ln(1+∂_*j*_/1 − ∂_*j*_) where ∂_*j*_=(1/*N*)∑_*n*_^1^*γWt*_*j*_(*n*)*H*_*j*_(*x*_*n*_) and *γ* = \{−1 if actual ≠ predicted 1, if actual = predicted.

Weight update equation for AdaCost, CSE_4_, and CSE_5_ is as follows:

(5) $$\begin{array}{c} Wt_{\left(j+1\right)}\left(m\right)=Wt_{j}\left(m\right)\exp\left(-\gamma \;H_{j}\left(x_{m}\right)\beta_{j_{{(\rangle }_{\gamma }}}\right). \end{array}$$

Here, *β*_*j*_ is identical in CSE_1_, CSE_2_, CSE_3_, and AdaBoost, whereas for AdaCost and CSE_4_ ∂_*j*_=(1/*N*)∑_*n*_^1^*γWt*_*j*_(*n*)*H*_*j*_(*x*_*n*_)*τ*_*j*_, where *τ*+*β* − =*C*_*n*_ for CSE_4_ and *τ*+=−0.5*C*_*n*_+0.5 and *τ* − =0.5*C*_*n*_+0.5 for AdaCost and CSE_5_. Furthermore, CSE_5_ does not include ϱ_*γ*_ in the calculation of ∂_*j*_ [33]. From the above weight update algorithmic equation, it has been noticed that the cost parameter is directly applied to all kinds of misclassification error (false-positive and false-negative) equally in each boosting round. They all have given equal weight to reduce cumulative misclassification costs. Table 1 depicts the summary of the survey for ten cost-sensitive boosting algorithms.

## 3. Proposed Clairvoyant Method

Different methodologies have been studied, and the most appropriate one is selected for this paper. In practice, there have been two schools of thought while dealing with misclassification costs. The first addresses the cost sensitizing with preprocessing the data by implementing various sampling techniques to increase the influence of the desired samples. These preprocessing techniques rely on examples in the training dataset to minimize cost. The second school of thought i to handle the problem more directly by building cost-sensitive adjustments into the algorithmic step. In this approach, the wealth of existing machine learning algorithms is modified to use the cost matrix. This mechanism gained significant popularity and became more demanding in practice. In the case of the second methodology, for example, AdaBoost and AdaCost, the metaclassifiers are extended to incorporate the cost of misclassification in the weight update method [34]. AdaBoost is a statistical classification meta-algorithm known for adaptive boosting, and it tweaks the learners in favour of instances misclassified by the previous classifiers. On the contrary, AdaCost is a misclassification cost-sensitive boosting method, a variant of AdaBoost. AdaBoostWithCost is an ensemble of AdaBoost and AdaCost to improve the performance. In this paper, the proposed algorithm belongs to the second methodology described above.

### 3.1. AdaBoostWithCost

Nonetheless, misclassification cost is not used in AdaBoost's weight update rule. In many other methods, the weight-updating rule increases the weights of wrong classifications more aggressively by applying the constant misclassification cost directly to the all misclassification errors (both false-positive and false-negative) equally in each boosting round. Such a traditional framework assumes that all misclassification errors carry the same cost. The proposed AdaBoostWithCost method applies the misclassification cost more specifically to the costly high-risk errors (false-negative in telecom churn study) instead of applying a constant cost to all misclassification errors directly in each iteration of boosting. The algorithm focuses on class-dependent cost sensitivity. The cumulative misclassification costs are reduced by assigning higher weights to costly high-risk errors over low-risk errors. The proposed new algorithm AdaBoostWithCost is illustrated in Algorithm 1.

### 3.2. Definitions of Symbols

All mathematical symbols and parameters used in equations of the proposed AdaBoostWithCost algorithm (described above) and flowchart shown in Figure 1 are described in Table 2. The description of the inventive steps is as follows. The central idea of the proposed AdaBoostWithCost algorithm is to increase the weight of the costly misclassified data points more aggressively than the correctly classified data points. Hence, the weight-updating rule increases the weights of the false negatives more than false positives since the false-negative error is more significant in the telecom churn prediction. In the above AdaBoostWithCost algorithm, steps 7 and 12 constitute the invented steps of the proposed AdaBoostWithCost algorithm. The weight update equation in each boosting round of AdaBoostWithCost is as follows:

(6) $$\begin{array}{c} P_{D\left(t+1\right)}\left(x_{i}\right)=\frac{P_{Dt}\left(x_{i}\right)\left(e^{-\alpha_{t}y_{i}h_{t}\left(x_{i}\right)+\left(-\gamma_{t}\right)C_{fn}y_{i}h_{t}\left(x_{i}\right)}\right)}{Z_{t}}. \end{array}$$

In the above equation, *P*_*D*(*t*+1)_ denotes the new probability assigned to the *i*^th^ data point *x*_*i*_ at (*t*+1)^th^ iteration and *P*_*Dt*_(*x*_*i*_) represents the distribution of *i*^th^ data point *x*_*i*_ at iteration *t*. The exponential loss function in the weight update equation is denoted by *e*^−*α*_*t*_*y*_*i*_*h*_*t*_(*x*_*i*_)+(−*γ*_*t*_)*C*_*fn*_*y*_*i*_*h*_*t*_(*x*_*i*_)^ consisting of two components or subexpressions as follows:

1. The first subexpression is −*α*_*t*_*y*_*i*_*h*_*t*_(*x*_*i*_)
2. The second subexpression which involves cost and false-negative misclassification error is (−*γ*_*t*_)*C*_*fn*_*y*_*i*_*h*_*t*_(*x*_*i*_)

It is worth mentioning that the value of the expression *y*_*i*_*h*_*t*_(*x*_*i*_) will be positive if *y*_*i*_*h*_*t*_(*x*_*i*_) is negative because the negative sign at the beginning changes negative *y*_*i*_*h*_*t*_(*x*_*i*_) to positive (since *α*_*t*_ is always positive). To elaborate more, in case of any misclassification performed by the model, the expression *y*_*i*_*h*_*t*_(*x*_*i*_) becomes positive, whereas in case of correct classification *y*_*i*_*h*_*t*_(*x*_*i*_) becomes negative. To more understand the reweighting formula, consider the case of a misclassification where *y*_*i*_*h*_*t*_(*x*_*i*_)=−1 (wrong prediction); hence, expression −*α*_*t*_*y*_*i*_*h*_*t*_(*x*_*i*_) is positive because always *α*_*t*_ > 0. Similarly, in case of accurate prediction, *y*_*i*_*h*_*t*_(*x*_*i*_)=+1 (correct prediction); hence, expression *y*_*i*_*h*_*t*_(*x*_*i*_) becomes negative according to the logic prescribed above. Therefore, the first subexpression −*α*_*t*_*y*_*i*_*h*_*t*_(*x*_*i*_) is exactly similar to AdaBoost's weight update equation and it can be derived from the above logic that AdaBoost boosts up the weights of the data points which have been misclassified consistently by earlier models and brings down the weight of the data points which have been classified correctly so that in the algorithm can focus more on the misclassified samples in its subsequent iterations. Nonetheless, the second subexpression (−*γ*_*t*_)*C*_*fn*_*y*_*i*_*h*_*t*_(*x*_*i*_) incorporates cost *C*_*fn*_ derived from the supplied cost matrix (described in Section 3.1) and the parameter *γ*_*t*_ which represents false-negative error at *t*_th_ iteration (on the contrary *α*_*t*_ is the total misclassification error used in the first subexpression). In the subexpression (−*γ*_*t*_)*C*_*fn*_*y*_*i*_*h*_*t*_(*x*_*i*_), the cost computation component is (−*γ*_*t*_)*C*_*fn*_. The other component *y*_*i*_*h*_*t*_(*x*_*i*_) holds the same evaluation method as described in the explanation of first subexpression. Hence, the subexpression (−*γ*_*t*_)*C*_*fn*_*y*_*i*_*h*_*t*_(*x*_*i*_) will be positive if the *y*_*i*_*h*_*t*_(*x*_*i*_) is negative because the negative sign at the beginning changes negative *y*_*i*_*h*_*t*_(*x*_*i*_) to positive and it is multiplied by cost *C*_*fn*_ for the false-negative error (denoted by *γ*_*t*_). Here, it is worth mentioning that since both *γ*_*t*_ and *C*_*fn*_ are always positive, the sign of entire expression (−*γ*_*t*_)*C*_*fn*_*y*_*i*_*h*_*t*_(*x*_*i*_) depends on the sign of *y*_*i*_*h*_*t*_(*x*_*i*_) as described above.

Therefore, in the second subexpression (−*γ*_*t*_)*C*_*fn*_*y*_*i*_*h*_*t*_(*x*_*i*_), the multiplication of cost *C*_*fn*_ to *y*_*i*_*h*_*t*_(*x*_*i*_) specifically for false-negative error (denoted by *γ*_*t*_) is the nucleus of the inventive step. The central idea of AdaBoostWithCost is to incorporate the extra cost specifically for false-negative error to enhance the boosting of the weight, in addition to the normal weight update performed by AdaBoost. This second subexpression underlines the fact that, to reduce the misclassification costs, costly and high-risk errors have been given more higher weights with respect to low-risk error. In short, in the AdaBoostWithCost algorithm, the weight-updating rule increases the weights of costly misclassified samples more aggressively than the correctly classified samples. The flowchart for AdaBoostWithCost is depicted below. In the flowchart, the inventive step of AdaBoostWithCost is specifically highlighted to demonstrate how AdaBoostWithCost incorporated the cost into the reweighting equation.  Table 3 demonstrates the key difference between their weight update equations.

### 3.3. Empirical Evaluation Parameters

The choice of measurement indices is of paramount importance to evaluate the classifier's performance. Different performance metrics are used to evaluate different classification algorithms. In the context of the current study, the false-negative classification error plays a pivotal role in telecom churn prediction. Thus, the study seriously focuses on the false-negative error counts for the empirical evaluation. The study also considers evaluating the other two parameters: misclassification cost and mean misclassification cost, which too holds great influence in the context of this study. The performance metrics are used to evaluate the performance of the proposed cost-sensitive boosting algorithm AdaBoostWithCost and AdaBoost. The cost of each class error is shown in the confusion matrix in Table 4, which is supplied as an input to measure the total misclassification cost. The normalized weight distribution concerning cost is shown in Table 5. More details about the confusion matrix and weight normalization method are stipulated in Section 3.1.

## 4. Empirical Evaluation

### 4.1. Data Selection

The telecom dataset used in the investigations has been taken from Kaggle [35]. The dataset contains over 3335 rows (Call Data Records) and 21 columns (attributes). Data consist of the various behaviours of customers, and the last column states if the customer is still with the existing telecom company or not. However, the study requires generating synthetic data (over 100,000 samples) to carry out the study's objective.

### 4.2. Generating Synthesized Data

The objective of the study's experiment is to empirically evaluate the performance of the proposed classifier AdaBoostWithCost with a large volume of data. Therefore, it enforces the study to generate synthesized data to fulfil the requirement for the investigation. The idea is to generate enough synthesized data (near about 100,000 samples) points, that is, Call Data Records (CDR), to compare the robustness of the AdaBoostWithCost method against discrete AdaBoost. The number of features in the Kaggle dataset is 21 features as well as only 3335 Call Data Records (CDR), which is not sufficient for satisfying the study's objective. Hence, it is essential to generate synthetic data from the source data collected from the Kaggle source. The synthetic data is generated by oversampling the source data using Weka [33] which transforms the source examples (data points) from 3335 CDR observations to 100,000 CDR observations that are adequate to satisfy the objective of the investigations.

### 4.3. The Input Cost Matrix and Weight Normalizations

Cost-sensitive machine learning methods explicitly use the confusion matrix as an input while building cost-sensitive classifiers. Fundamentally the cost matrix is a matrix that assigns a cost to each cell in the confusion matrix. The effectiveness of cost-sensitive learning relies strongly on the supplied cost matrix. Parameters provided in the confusion matrix have the utmost importance in both training and prediction steps [36] in the study of cost-sensitive learning. In most of the cost-sensitive boosting algorithms, the cost matrix is supplied in the model-building phase. The cost-sensitive boosting classifiers modify the weight update equation to incorporate the misclassification cost derived from the cost matrix. Defining the confusion matrix might sometimes be challenging as it is domain-specific. In the telecom churn prediction modeling study, a model is used to predict which customers are more likely to abandon a service provider. In this context of the study, failing to detect an actual churning customer (false-negative case) has a more serious impact on economic results than failing to identify accurately a nonchurning customer (false-positive case). Hence, in this study, the proposed cost-sensitive boosting algorithm specifically focuses on reducing cumulative high-risk misclassification error (false-negative), and, accordingly, the confusion matrix parameters are defined.

Ideally, an accurate cost matrix might be correctly defined by a domain expert or economist. In this study, since the incorrect prediction of the churning customer (false-negative) has bigger influence, the proposed AdaBoostWithCost algorithm focuses on reducing specifically high-risk costly errors. Regarding the allocation of the cost for each class in the cost, the matrix is shown in Table 6. It has been observed by most telecom experts from various literature surveys that false-negative classification error is 5 to 10 times more expensive than false-positive error. Considering a worst-case scenario in telecom industries, this study assigns the false-negative cost ten times (extreme case) more than the false-positive cost. Hence, the cost ratio of false-positive errors to false-negative errors used in this study is 1 : 10, which means that false-negative errors are ten times costlier than the false-positive classification errors. The study experiments with running three different sets of iterations for empirical evaluation of AdaBoostWithCost and AdaBoost. It is important to note that Table 4 depicts a hypothetical cost matrix supplied as an input to the AdaBoostWithCost algorithm and used in the weight update equation to calculate the misclassification cost. In the below cost matrix, in Table 4, the notation *C* () indicates the cost. In *C* (*x*, *y*), the first parameter *x* is the predicted class, and the second parameter *y* represents the actual class. Table 4 represents the confusion matrix; the names of each cell of the confusion matrix are also listed as acronyms; for example, false positive is FP. Table 4 shows the cost-matrix structure where the cost of a false positive is denoted by *C*(1, 0) and the cost of a false negative is denoted by *C*(0, 1).

Table 6 depicts the cost matrix which is supplied as input to the AdaBoostWithCost algorithm and used in the weight update equation. The assignment of a cost to each cell in the confusion matrix is defined below and referred to as the confusion matrix. It is noteworthy that cell *C*(0, 1) of the confusion matrix represents the cost of false-negative error, whereas false-positive error is designated by cell *C* (1, 0). Consequently, cell *C* (0, 1) is assigned to cost 10, and cell *C* (1, 0) is assigned to 1 according to the aforementioned discussion (the study considers that the false-negative error is 10 times more costly than the false-positive error). Table 6 shows each cell value of the confusion matrix.

Although the confusion matrix consists with four cells, nevertheless, the true positive and true negative do not play an important role in the context of telecom churn prediction. Moreover, false-positive classification has also an insignificant impact on the context of the study. The only significant parameter is false-negative classification which has a serious impact in telecom churn modeling, hence the high value of 10 assigned to cell *C* (0, 1). The calibration of weight distribution with respect to cost is essential to carry out the weight update step in AdaBoostWithCost. The normalization (rescaling) method to transform false-negative value to weight distribution is mentioned in Table 5. To use the cost matrix in the proposed classifier, the confusion matrix cell values must be rescaled within the range of 0 to 1. This normalization or calibration [37] is an essential step to perform the weight update operation in the reweighting equation of the AdaBoostWithCost algorithm. The normalization technique ensures that the weight or probability distribution of each training data point stands between 0 and 1. The investigation of this study centered around false-negative cost 10 and corresponding weight distribution 0.2, highlighted in Table 5.

### 4.4. Experimental Method

The investigations of the study estimate the three measure indices for telecom churn prediction which have utmost importance, the false-negative errors, misclassification cost, and mean misclassification cost, to assess the performance of the proposed AdaBoostWithCost classifier. The empirical evaluation of this study demonstrates two significant aspects of benchmarking the performance of the AdaBoostWithCost algorithm against AdaBoost. First, the study focuses on measuring performance metrics: the false-negative errors, misclassification cost, and mean misclassification cost (average misclassification costs across all sets of iterations). Second, it graphically plots the misclassification error rate (both training and test error rates) concerning multiple boosting rounds. To carry out the second measurement criteria mentioned above, this study computes the training and test misclassification error rates for each boosting round of the proposed AdaBoostWithCost classifier and plots them graphically to demonstrate the performance curve of AdaBoostWithCost boosting classifier and basic AdaBoost classifier. The input cost matrix for each category of errors is defined in Table 4. Here, it is important to mention that false-negative error observation is the foremost interest in this study, since it significantly impacts revenue generation in telecom churn prediction. The false-positive errors are not accounted for seriously in the experiment, since they are insignificant compared to false-negative errors in this context.

Literature states that false-negative classification error is generally 5–10 times more costly than the false-positive classification error in telecom churn modeling. This study considered the worst-case scenario of the telecom industry, that is, presumed the most severe impact on the revenue generation for service providers due to the incorrect false-negative classification. Given this worst-case scenario, the experiment assigns the false-negative cost ten times (highest possible impact on business) more than the false-positive cost. It is to be noted that cell *C* (0, 1) of the confusion matrix represents the cost of false-negative errors, whereas false-positive error is designated by cell *C* (1, 0). Consequently, cell *C* (0, 1) is assigned to cost 10, and cell *C* (1, 0) is assigned to 1. While estimating the three critical performance metrics, the cost matrix must be rescaled or normalized to a range of 0 to 1. This normalization of probability calibration [37] is mandatory to execute the weight update operation in the reweighting equation of the AdaBoostWithCost algorithm as the weight (probability) distribution of each data point varies between 0 and 1. The normalization method for transforming the confusion matrix's false-negative value to weight distribution is mentioned in Table 5.

The first aspect of the empirical evaluation illustrated above is to determine by using three sets of iterations 10, 20, and 40 to measure the performance metrics; the false-negative errors, misclassification cost, and mean misclassification cost are explained as follows: the misclassification cost for each set of iterations (10, 20, and 40 used in the experiment) of the AdaBoostWithCost algorithm is computed from the following formula:

(7) $$\begin{array}{c} \text{the misclassification cost}=\text{CM}\left[C\left(0,1\right)\times \text{false negatives}+C\left(1,0\right)\times \text{false positives}\right], \end{array}$$

where **CM** is the confusion matrix and **C** (row_index, col_index) is the cost of the cell.

The study uses iteration-wise computation of cumulative misclassification cost:

- Cumulative misclassification cost at the end of the 10^th^ iteration
- Cumulative misclassification cost at the end of the 20^th^ iteration
- Cumulative misclassification cost at the end of the 40^th^ iteration

The misclassification cost is determined by the following formula: mean misclassification cost = cumulative misclassification cost of all iterations over the number of a set of iterations.

(8) $$\begin{array}{c} \text{Mean misclassification cost}\approx \frac{\left(a+b+c\right)}{3}, \end{array}$$

where *a*, *b*, and *c* are the above steps to calculate the misclassification cost resulting from each set of iterations, and there are three sets of iterations (10, 20, and 40) that have been used for the experiment to compute the mean misclassification cost. The second aspect of the empirical evaluation specified above is to visually represent the misclassification error rate for both training and test errors by plotting graphs. One of the salient features of the investigation is to manifest the change in training and test error rate over each set of boosting rounds.

## 5. Results and Discussion

### 5.1. The Evaluation of AdaBoostWithCost and AdaBoost

The error summary of the experimental results focuses on the three important performance metrics: the total misclassification error, false-negative error count, and training and testing error rates. Upon careful inspection of the below synopsis, it is obvious that the values of three performance metrics consistently decrease over each set of boosting rounds 10, 20, and 40, respectively. Specifically, the false-negative error, which is a parameter of utmost importance in this study, gets reduced significantly over each interval of boosting rounds.

### 5.2. Interpretation of Empirical Results and Visualizations

The empirical evaluation of the proposed AdaBoostWithCost algorithm and AdaBoost classifier has been carried out in three crucial performance metrics considered in the study context. The summarized error summary is shown in Table 7. Table 7 manifests the significant difference in experimental results between AdaBoostWithCost and AdaBoost. The study observed that AdaBoostWithCost significantly reduced the false-negative error counts compared to the traditional boosting classifier AdaBoost. Hence, the summarized results unfold the fact that AdaBoostWithCost prevails over AdaBoost in terms of false-negative error reduction, which is the foremost influential parameter in the context of the study.

Figure 2 demonstrates how misclassification error rates of both classifiers monotonically decrease with the increasing number of iterations. Nevertheless, the span of the sharp falling edge shown as the dark blue line (indicating AdaBoostWithCost) unveils the fact that the pace of error rate reduction by AdaBoostWithCost is more expeditious than that by traditional AdaBoost. Figure 2 also reveals eventually that AdaBoostWithCost beats AdaBoost in the race of error rate reduction. The below side-by-side graph shows the decreasing pattern of training and test rates with each set of iterations for both AdaBoost and AdaBoostWithCost classifiers. The above plots show how both training and test error rates gradually get scaled down over each iteration round. Moreover, the line graphs portray how the training and test error rates monotonically decrease when the number of iterations is increased. By careful inspection, the study discovers that the intermediate gap between the two lines (training and test error rates) demonstrates that training and test error rates reduction is much expedited by AdaBoostWithCost compared to the traditional AdaBoost classifier. The study also concludes from Figure 3 that the AdaBoostWithCost model does not tend to overfit. However, there is a chance of slight overfitting in the case of AdaBoost classier.

## 6. Conclusion

Cost-sensitive learning is not new in today's machine learning community. In recent years, it has gained tremendous popularity because of the rising demand for critical real-world cost-sensitive applications. Today, state-of-the-art machine learning algorithms are not well designed with financial goals, in the sense that the models miss including the real financial costs during the training and evaluation phases. In the context of telecom churn prediction, a model evaluation based on a traditional measure such as accuracy does not yield the best results when measured by the actual financial cost. Failing to detect true churners severely impacts telecom operators' revenue rather than incorrectly predicting a nonchurning customer as a churner. This paper intended to deal with the challenges of class-dependent cost-sensitive classification and mitigate the business-specific cost sensitivity. This paper surveyed various cost-sensitive boosting algorithms in today's machine learning community and summarized their comparison in Table 1. The study also discussed the weight update equation of those cost-sensitive classifiers while dealing with variable cost errors. Nevertheless, the study significantly contributed to class-dependent cost-sensitive boosting classification in two distinct aspects: First, the study devised a novel class-dependent cost-sensitive boosting algorithm, AdaBoostWithCost, which incorporates the cost function into the weight update equation in a novel way. The inventive step of AdaBoostWithCost is in the weight update equation, which incorporates the unique cost function. The AdaBoostWithCost classifier applied the misclassification cost in the reweighting equation more specifically to the high-risk errors (false-negative error in the telecom churn case) instead of applying to all misclassification errors directly in each iteration of boosting. Second, the study carried out an in-depth inspection of experimental results summarized in Table 7 and the interpretation of graph visualizations (Figures 2 and 3). Finally, the study has drawn a significant conclusion that the AdaBoostWithCost algorithm consistently outperforms AdaBoost in all aspects of the study's objective.

## Figures and Tables

**Figure 1:** The flowchart of the AdaBoostWithCost algorithm.

**Figure 2:** The total misclassification error rate of AdaBoostWithCost versus AdaBoost.

**Figure 3:** Training and test error rates of AdaBoost versus AdaBoostWithCost.

**Algorithm 1:** AdaBoostWithCost: the proposed cost-sensitive boosting algorithm.

**Table 1:** Comparison of cost-sensitive boosting algorithms.

Classifiers	Initial weight distribution	Is class-dependent cost-sensitive?	Reweighting used?^*∗∗*^
Boosting	1/*N*	No	No
Cost-Boost	1/*N*	No	Yes#
Uboost	(Unequal)^$^	No	No
Cost-Uboost	(Unequal)^$^	No	Yes^#^
AdaBoost	1/*N* (Equal)	No	No
AdaCost	1/*N* (Equal)	Yes	Yes
CSE_1_	Equal	No	Yes^#^
CSE_2_	Equal	No	Yes^#^
CSE_3_	Equal	No	Yes^#^
CSE_4_	Equal	No	Yes^#^
CSE_5_	Equal	No	Yes^#^

$ = initial weights: *w*(*m*)=*w*^*i*^=*c*^*i*^(*N*/Σ_*I*_*C*^*j*^*N*^*j*^), ^∗∗^=reweighting rules: updated new weight = cost of misclassification; ^*∗*^ old weight (if wrongly classified); new weight = old weight (if correctly classified); # = algorithm specific weight update equation.

**Table 2:** Definitions of symbols of the equations.

H	Final hypothesis/model combining all weak hypotheses
*h*_*t*_	The hypothesis/model at *t*^th^ iterations
*h*_*t*_(*x*_*i*_)	The prediction of the *t*^th^ data point *x*_*i*_ by the hypothesis/model *h*_*t*_
*P*_*Dt*_(*x*_*i*_)	The probability distribution of the *t*^th^ data point *x*_*i*_
*P*_*D*(*t*+1)_	The new probability of the *i*^th^ data point *x*_*i*_ at (*t*+1)^th^ iteration
*α*_*t*_	Hypothesis's weight for gross misclassification error at *t*^th^ iteration
*γ*_*t*_	Hypothesis's weight for high-risk (false-negative) error at *t*^th^ iteration
*C*_*fn*_	Cost of misclassification for false-negative error specified in the input cost matrix
*y*_*i*_	$\left\{\begin{array}{cc} -1, & \text{if actual}\neq \text{predicted},\\ 1, & \text{if actual}=\text{predicted}. \end{array}\right)$
*Z*_*t*_	∑_*i*=1_^*n*^*P*_*Dt*_(*x*_*i*_)(*e*^−*y*_*i*_*h*_*t*_(*x*_*i*_)(*α*_*t*_+*β*_*t*_*C*_*fn*_)^), the normalization

**Table 3:** Reweighting step of discrete AdaBoost and proposed AdaBoostWithCost.

Discrete AdaBoost	AdaBoostWithCost
Update weight step:	Update weight step:
*P*_*D*(*t*+1)_=*P*_*D*_(*x*_*i*_)(*e*^*α*_*t*_*y*_*i*_*h*_*t*_(*x*_*i*_)^)/*Z*_*t*_	*P*_*D*(*t*+1)_=*P*_*D*_(*x*_*i*_)
	(where *Z*_*t*_=∑_*i*=1_^*n*^*P*_*Dt*_(*x*_*i*_)(*e*^*α*_*t*_*y*_*i*_*h*_*t*_(*x*_*i*_)^))

(*e*^−*α*_*t*_*y*_*i*_*h*_*t*_(*x*_*i*_)+(−*γ*_*t*_)*C*_*fn*_*y*_*i*_*h*_*t*_(*x*_*i*_)^)/*Z*_*t*_	≈*P*_*D*(*t*+1)_=*P*_*D*_(*x*_*i*_)(*e*^−*y*_*i*_*h*_*t*_(*x*_*i*_)(*α*_*t*_+*γ*_*t*_*C*_*fn*_)^)
	(where *Z*_*t*_=∑_*i*=1_^*n*^*P*_*Dt*_(*x*_*i*_)(*e*^−*y*_*i*_*h*_*t*_(*x*_*i*_)(*α*_*t*_+*γ*_*t*_*C*_*fn*_)^))

*P*_*D*(*t*+1)_ is the new probability assigned to the *i*^th^ data point *x*_*i*_ at (*t*+1)^th^ iteration; all other parameters constituting the right side of the equation are described as follows: *α*_*t*_ = hypopaper's weight for gross misclassification error at *t*^th^ iteration, *γ*_*t*_ = false-negative error at *t*^th^ iteration, *C*_*fn*_ = misclassification cost for false-negative error specified in the input cost matrix,$\text{where},\left\{\begin{array}{cc} -1, & \text{if actual}\neq \text{predicted}\\ 1, & \text{if actual}=\text{predicted} \end{array}\right)$.

**Table 4:** The confusion matrix.

	Actual negative	Actual positive
Predicted negative	*C*(0, 0) TN	*C*(0, 1) FN
Predicted positive	*C*(1, 0) FP	*C*(1, 1) TP

**Table 5:** The weight normalization matrix.

Cost of false negatives	5	10	20	40	80	100
Weight distribution	0.1	0.2	0.4	0.6	0.8	1

**Table 6:** Cost assignment to confusion matrix.

	Actual negative	Actual positive
Predicted negative	0	10
Predicted positive	1	0

**Table 7:** Summarized comparison of measure indices.

Iteration rounds	Performance metrices	AdaBoost classifier	AdaBoostWithCost classifier
10	False-negative error	649	388
	Misclassification cost	8422	7015

20	False-negative error	463	345
	Misclassification cost	7036	6802

40	False-negative error	390	70
	Misclassification cost	6521	5168

Mean misclassification cost		6676.3	6328.3

## Data Availability

The data used to support the findings of this study are available from the corresponding author upon request.
